The article "Cervical Lesion Classification Method Based on Cross-Validation Decision Fusion Method of Vision Transformer and DenseNet" was published in 2022. Journal: J Healthc Eng.

# Cervical Lesion Classification Method Based on Cross-Validation Decision Fusion Method of Vision Transformer and DenseNet

**DOI:** 10.1155/2022/3241422

**Published:** 2022-05-14

**Authors:** Ping Li, Xiaoxia Wang, Peizhong Liu, Tianxiang Xu, Pengming Sun, Binhua Dong, Huifeng Xue

**Affiliations:** ^1^Department of Gynecology and Obstetrics, Quanzhou First Hospital Affiliated to Fujian Medical University, Quanzhou 362000, Fujian, China; ^2^School of Medicine, Huaqiao University, Quanzhou 362000, Fujian, China; ^3^College of Engineering, Huaqiao University, Quanzhou 362000, Fujian, China; ^4^Fujian Maternity and Child Health Hospital, Affiliated Hospital of Fujian Medical University, Fuzhou 350001, Fujian, China

## Abstract

**Objective:**

In order to better adapt to clinical applications, this paper proposes a cross-validation decision-making fusion method of Vision Transformer and DenseNet161.

**Methods:**

The dataset is the most critical acetic acid image for clinical diagnosis, and the SR areas are processed by a specific method. Then, the Vision Transformer and DenseNet161 models are trained by the fivefold cross-validation method, and the fivefold prediction results corresponding to the two models are fused by different weights. Finally, the five fused results are averaged to obtain the category with the highest probability.

**Results:**

The results show that the fusion method in this paper reaches an accuracy rate of 68% for the four classifications of cervical lesions.

**Conclusions:**

It is more suitable for clinical environments, effectively reducing the missed detection rate and ensuring the life and health of patients.

## 1. Introduction

Cervical cancer is the fourth most common female cancer in the world, which seriously threatens women's health [1]. Pathological studies of cervical cancer have shown that persistent infection of high-risk human papillomavirus (HPV) is the main cause of the occurrence and development of cervical lesions and cervical cancer. During this period, infected patients will experience a long period of precancerous lesions, which are divided into three stages: CIN1, CIN2, and CIN3 according to the severity [2], as shown in Figure 1. Clinicians have sufficient time to make a diagnosis. Through early diagnosis and early detection, morbidity and mortality can be greatly reduced, and the survival period can be prolonged. At present, the mainstream screening methods are Pap smear, HPV test, and colposcopy [3]. Among them, colposcopy has become the first choice in resource-poor areas due to its simple operation, low cost, and relatively noninvasive advantages. However, as an optical instrument, its diagnostic results are highly subjective and low in specificity, and there is the possibility of missed diagnosis and misdiagnosis.

In recent years, with the rapid development of artificial intelligence (AI) technology, deep learning has made a breakthrough in the field of medical image processing [4], including MR images [5], CT images [6], and histopathological images [7], which is helpful for the detection and diagnosis of cancer [8]. Similarly, deep learning also provides new ideas for colposcopy image analysis. But at the same time, there are still some problems that need to be better solved. The specular reflection (SR) areas are very similar to the lesion area after adding acetic acid, which interferes with the diagnosis. In addition, there is little difference between several lesion grades in the image, and it is difficult to classify them [9]. Most researches focus on the exploration of the dichotomy of CIN2+. Therefore, this paper studies the risk assessment method of cervical lesions based on colposcopy images. After the SR area processing, the images treated with acetic acid are classified by multimodel fusion, and the corresponding clinical assessment is made.

## 2. Related Work

### 2.1. Cervical Lesion Classification

For the classification of cervical lesions in colposcopy images, the lesion feature information that traditional methods pay attention to mainly includes texture and color. For example, Kim and Huang [10] extracted the color and texture features of large batches of cervical images as feature training libraries and trained a classic SVM classifier for classification. In addition, Li and Poirson [11] analyzed the features of abnormal blood vessels in cervical lesions, while Park et al. [12] paid attention to the spatial correlation of lesion features in cervical images. The more mature research is the series of work of Xu et al. [13, 14], which deeply extracts features from three types of features: the pyramid histogram of oriented gradients (PHOGs), the pyramid color histogram in LAB space (PLAB), and the pyramid histogram of the local binary pattern (PLBP). Song et al. [15] also used expert-annotated handcrafted features combined with clinical diagnosis results for cervical lesion classification. Other researchers [16] focus on the combination of multiple reagent images during colposcopy to extract the color and texture features of the lesion area. However, whether it is based on the feature extraction of various images or the manual annotation features of experts, traditional auxiliary diagnosis methods focus on low-dimensional features of images, and the feature classification methods that are highly dependent on manual selection have limited practical significance in the clinical promotion.

Therefore, with the rapid development of AI, researchers applied it to the classification of cervical lesions for colposcopy image analysis and constantly explored and excavated the deep features of cervical images. One is to directly apply the mature deep convolutional network in the field of computer vision to the classification of cervical lesions in colposcopy images. For example, Xu et al. [17, 18] used a pretrained AlexNet network to classify the types of cervical dysplasia, Hu et al. [19] and Chen [20] et al. used the Faster R-CNN model to effectively detect cervical lesion regions, and Zhang et al. [21] proposed a fine-tuned classification model of cervical lesions with densely connected neural network DenseNet121. Another is to modify the existing model for colposcopy images to improve the accuracy of cervical lesion diagnosis. On the one hand, there are some studies on the improvement of a single model, such as ColpoNet--a classification architecture of cervical cancer based on self-learning ability [22], the image classification of cervical lesions based on regularized transfer learning strategy [23], convolutional neural network recognition based on CapsNet for cervical lesions classification [24], and the integrated CAIADS model of cervical lesion classification and detection [25]. On the other hand, there are two common decision-making methods combining the features of convolutional neural networks: Yuan et al. [26] used ResNet to classify the lesion level, segmented the lesion area through U-net, and combined Mask R-CNN for final detection; Cho et al. [27] combined two network models, Inception and ResNet, to classify lesions; Luo et al. [28] optimized the output of the two models, RseNet50 and DenseNet121, through the strategy of decision feature integration and fusion; Elakkiya et al. [29] put forward the FSOD-GAN model combining FR-CNN, GAN, and FSDAE technologies. A newer study also combined convolutional neural networks with clinical features of cervical lesions [30].

Compared with the clinician's manual reading and traditional CAD methods, the introduction of AI makes the diagnosis of cervical lesions in colposcopy images achieve better results. However, few of these studies are used in clinical practice. One of the main reasons is that they mostly focus on the dichotomous studies of CIN2+ or HSIL+, which are not suitable for clinical screening in the actual process. In addition, there is less processing for the SR areas of colposcopy images, which will interfere with classification and diagnosis to a certain extent.

### 2.2. Transformer

Transformer [31] was published by Google on Computation and Language in 2017. It was originally proposed for the field of Natural Language Processing (NLP). Before that, Recurrent Neural Network (RNN) model had limited memory length and could not be parallelized, but Transformer realized this function and achieved great success in the field of NLP. However, after the DEtection TRansformer (DETR) algorithm [32] applied Transformer to the object detection task in computer vision and achieved excellent performance, Transformer also began to attract attention in the field of computer vision (CV).

Studies have shown that Transformer is not only suitable for high-level tasks such as image classification, object detection, and lane detection but also has made breakthroughs progress in low-level tasks such as image augmentation. There is no doubt that Transformer is one of the most noteworthy directions in the field of CV at present.

### 2.3. Fusion

Without changing the model, it is a simple but effective fusion method to directly vote or average the final predicted results of different models. But the precondition is that the models are independent of each other, and there is no strong correlation between the results. The greater the correlation difference between the models, the better the fusion effect will be.

At present, in the classification study of cervical lesions based on colposcopy images, multiple deep convolutional neural network (CNN) models are used for training in model fusion [28, 29]. The core of the deep CNN lies in each convolutional layer. The low-dimensional convolutional layer generally learns more prominent feature information such as image texture, while the high-dimensional convolutional layer focuses more on the more abstract global information in the image. Although there are certain differences in the final features extracted by different network structures, the mechanisms of feature extraction from various CNNs are similar.

## 3. Methodology

In this paper, acetic acid images, which are the most critical for clinical diagnosis, are adopted. Firstly, the overall generalization ability is increased by means of data augmentation. After experimental research, two models, Vision Transformer and DenseNet161, which have great differences in correlation, are selected for fivefold cross-validation. Then, the fivefold prediction results corresponding to the two models are fused by weights. Finally, the results are averaged to obtain the maximum probability value; that is, the corresponding lesion category is obtained. The overall scheme is shown in Figure 2.

### 3.1. Data Preprocessing

The data collected in the clinic are complicated and there is no uniform standard for the image format, so the computer cannot directly and effectively process them. At the same time, the particularity of medical image data makes it difficult to obtain in large quantities, so it is difficult to guarantee the amount of training data. Therefore, preprocessing the original data is the first step in the whole experiment.  Figure 3 shows the data preprocessing process of colposcopy data before training in this paper.

As shown in Figure 3, according to the clinicopathological results, the data were divided into four categories, namely, negative, LSIL, HSIL, and cancer. At the same time, the region of interest (ROI) of the image, that is, the clinical transformation zone (TZ), was obtained based on the cervical region labels labeled by experts. Then, the SR areas are removed by the specific method [33], and the processed images are uniformly standardized to 224 *∗* 224 for network training. Finally, the data augmentation method is used to increase the amount of training data, reduce overfitting, and increase the generalization ability of the model. The figure shows the augmented data generated by rotation (90 degrees), brightness (offset 30%), and contrast (offset 50%).

### 3.2. Vision Transformer Processing of Cervical Images

Vision Transformer was proposed by Dosovitskiy et al. [34] for the direct application of Transformer structure to image processing. An image is divided into multiple patches, similar to the words of NLP. The input is these patches after a series of linear embedding operations. The disadvantage of this method is that it may lack the inherent inductive biases of CNN, such as translation invariance and locality, which makes its generalization performance poor when there are few training sets. But at the same time, the authors found that the Vision Transformer can perform better by pretraining on a larger dataset and then transferring to other tasks. Therefore, we also adopted the weights obtained by pretraining on the ImageNet21K image dataset and applied them to our own cervical image data training after fine-tuning.

According to the idea of the original model, we trained the cervical image data by Vision Transformer, and its basic structure framework is shown in Figure 4.

Firstly, the cervical image is changed into a two-dimensional matrix required by the Transformer Encoder through an embedding layer. That is, each cervical image is divided into several patches according to a given size, and each patch is mapped to a one-dimensional vector by linear mapping. It is worth noting that before entering the Transformer Encoder, it is necessary to add the token and Position Embedding specially used for classification, which are stitched together with the tokens previously generated from the cervical image. The Position Embedding uses a trainable parameter that is directly superimposed on tokens, so the size should be consistent.

Then, enter the Transformer Encoder module. Each token is processed through Layer Norm, a normalization method. Two core parts are followed, one is to use the Multihead Attention mechanism to combine the image information learned from different parts and directly use the Dropout layer to alleviate the training overfitting. The other is an MLP Block consisting of a fully connected layer, GELU activation function, and Dropout. The whole constitutes the Encoder Block and repeatedly stacks the output *L* times.

Finally, the final classification prediction result is obtained through the MLP Head composed of linear layers. Note that what we get here are the probability values that the model predicts that a cervical image belongs to each of the four categories, respectively.

### 3.3. DenseNet161 Processing of Cervical Images

DenseNet [35] is an innovative work after condensing the most essential parts of ResNet [36], and its core idea lies in dense connections. DenseNet strengthens feature propagation, encourages feature reuse, and directly connects all inputs to the output layer, effectively alleviating the problem of gradient disappearance. At the same time, the use of dense block, Transition layer, and smaller growth rate makes the network narrower, which greatly reduces the number of parameters and effectively suppresses overfitting.

According to the basic structure of DenseNet161 [35], the process framework of cervical image data learning and training through DensNet161 is shown in Figure 5.

Similarly, the final classification prediction result is obtained by DenseNet161, that is, the probability values of the four categories predicted by the second fusion model for the same cervical image.

### 3.4. Fivefold Cross-Validation Decision Fusion

Different from the previous research on the fusion of multiple CNNs, we innovatively fuse the classification probabilities predicted by Vision Transformer and DenseNet161 for fivefold cross-validation decision fusion. The correlation between the two models is quite different, and more feature information in colposcopy images can be learned.

First of all, the transfer learning method is adopted to fine-tune Vision Transformer and DenseNet161 models through the weights obtained on the ImageNet dataset to get fivefold learning weights. Then, the *i*-fold prediction results corresponding to the two models are fused by weights, and the fusion method is defined as follows:

(1) $$\begin{array}{c} F_{i}=X_{\text{fusion}}\left(V_{i},D_{i}\right)=V_{i}\omega_{1}+D_{i}\omega_{2}. \end{array}$$

Here, *i* ∈ [1, 5], *X* is the fusion algorithm, and *V*_*i*_ and *D*_*i*_, respectively, represent the prediction results of the *i*th fold of Vision Transformer and DenseNet161. *ω*_1_ and *ω*_2_ represent different artificially set weights, and *F*_*i*_ is the *i*th fold of the two models. Finally, the average operation is performed on the obtained five fusion results to obtain the maximum probability; that is, the final lesion category is obtained, as shown in

(2) $$\begin{array}{c} R=\text{Avg}\left(F_{1},F_{2},...,F_{5}\right). \end{array}$$

Through the fivefold cross-validation decision fusion, the classification accuracy of cervical lesion images can be improved to a certain extent.

## 4. Experiments

In the experiment part, the dataset used in the experiment is first introduced, then the selected evaluation indicators are correspondingly explained, and finally, the experimental details and related results are displayed.

### 4.1. Dataset

The experimental data were collected from the colposcopy images of Fujian Maternal and Child Health Hospital from October 2016 to April 2018. Only the most critical acetic acid images in clinical diagnosis were selected for the experiment. The data of each subject included the data of acetic acid images and their corresponding pathological diagnosis results. The study included 732 subjects with a total of 2512 colposcopy images. The distribution of experimental data is shown in Table 1. Among them, 100 cases were selected for testing, and a total of 100 images were randomly selected from each case to form the test set. The remaining 2412 images were used for training and validation, and each category was roughly divided into five equal parts, which were mixed with one part of the other categories. This constituted the basic dataset of fivefold cross-validation; that is, the training set and the validation set are distributed according to the ratio of 4 : 1 for each epoch.

### 4.2. Evaluation Indicators

For the prediction results of cervical lesions in colposcopy images, we compared the diagnostic performance with the commonly used evaluation indicators in classification, including average accuracy (ACC), sensitivity (SEN), specificity (SPEC), positive predictive value (PPV), negative predicted value (NPV) [37], and F1-score value [38]. The relevant formula definitions of these five indicators are shown in Table 2, where TP, TN, FP, and FN are the numbers of true positive, true negative, false positive, and false negative in the diagnostic results of the test images, respectively. Among them, the F1 score is often used for imbalanced data classification to evaluate the comprehensive performance of classification models. However, the data of the HSIL category in our experiment is obviously higher than that of other categories, and there exists an imbalance between categories. Therefore, in this study, the evaluation of the classification model in colposcopy images pays more attention to the F1-score value on the basis of the comprehensive evaluation of various indicators.

### 4.3. Experimental Results

The experimental environment of this paper is Python3.8. The CPU is an Intel i7-8700K (3.20 GHz) and the memory is 8.00 GB. According to the experimental comparison, for our colposcopy image dataset, the optimization methods of Vision Transformer and DenseNet161 are both SGD algorithms. The initial learning rate and weight decay of the former are 1E-5 and 5E-5, while the latter is set to 1E-5 and 1E-4, respectively.

#### 4.3.1. Comparison with State-of-the-Art Methods

First, our fusion model is compared with several state-of-the-art models in the field of CV, including Vision Transformer [34], ShuffleNetV2 [39], MobileNetV3 [40], EfficientNetV2 [41], and DenseNet161 [35]. Note that the experimental method of Densenet161 here refers to [21], but the final prediction is refined into four categories consistent with the research in this paper. The model comparison results are shown in Table 3.

According to Table 3, it is found that ACC of the fusion method in this paper is the best, and the other indicators are basically ranked in the top. Especially for cancer, all indicators reached 90%. Here, we notice that among the compared models, Vision Transformer has the lowest prediction accuracy for a cervical lesion in colposcopy images, while DenseNet161 is the highest, with a slight advantage of 0.02 over the subsequent EfficientNetV2. At the same time, we also observed that MobileNetV3 has better prediction performance for the negative category, and F1 score, PPV, and SPEC are slightly higher than other models.

#### 4.3.2. Fusion Contrast

Next, we fuse several models in pairs according to the fusion idea in this paper. All the combined experimental results are shown in Table 4. In the table, *ω*_*1*_ and *ω*_*2*_ are the weight values of each model corresponding to the best accuracy after the two models are fused. Specifically, for a group of fusion experiments, the weights of the two models start from 0 to 1 simultaneously and then automatically increase or decrease by 0.05 each time. All experimental results shown in this table are the best after trying these weights.

Through experimental comparison, we found that the ACC of the DenseNet161 model after fusion with EfficientNetV2 and Vision Transformer is 0.68, ranking first. Therefore, aiming at the fusion of these two different models, we conducted a more detailed comparison.

Firstly, we compared the five major indicators except the accuracy, as shown in Table 5. It can be seen that the fusion of DenseNet161 and Vision Transformer has a slight advantage in CV evaluation, and the F1 value is better. In the case of imbalance between colposcopy image categories, the higher F1 value indicates that the model is less affected by differences in sample size, which is suitable for this particular dataset and clinical application environment.

Then, the specific prediction results of 100 test images are compared, and the confusion matrices of the two fusions are shown in Figures 6(a) and 6(b). Of the 100 images tested, the most difference between them is the prediction of the HSIL categories in one of them. The fusion of DenseNet161 and EfficientNetV2 is predicted to be negative, while the fusion of DenseNet161 and Vision Transformer is slightly better for predicting the HSIL category. This is also more suitable for the clinical application of the colposcopy image classification model. In the process of diagnosis, colposcopy physicians are more inclined to diagnose the images as high-level lesions in the face of images that are difficult to define and, further, make a definite diagnosis by pathological biopsy. Because lesion diagnosis is a special classification task, physicians hope to ensure a less missed diagnosis rate and are responsible for the patients' life and health.

#### 4.3.3. Clinical Comparison

Finally, we compared the fusion model with colposcopy physicians. We adopted a retrospective study, in which we extracted the clinician's diagnosis results from the patient's diagnosis report, and 100 test images corresponded one by one. The clinician's diagnosis results and the prediction results of the fusion model in this paper are compared with the pathological report, and TP, TN, FP, and FN are obtained, respectively. Then, the six evaluation indicators mentioned above are calculated. The comparison results for 100 test images are shown in Table 6. It can be seen that, on the average level of physicians, the ACC of our fusion model has improved by 6 points, and the F1 score values are higher than those of physicians. In addition, we communicated with physicians and analyzed the slightly lower data indicators in this experiment. We found that physicians' diagnosis is generally conservative, and they tend to take a higher level when diagnosing cervical lesions. Thus, the FN value is smaller, and the corresponding indicators would increase.

## 5. Limitation and Discussion

Related research shows that HPV testing has higher coverage and better age compliance than Pap smears in early cervical cancer screening [42]. Unlike these methods analyzed from the perspective of genetic testing and cytology, colposcopy is more intuitive to observe and diagnose from the morphology. Although all these mainstream methods have an important impact on the early diagnosis of cervical cancer, the expensive and time-consuming manual screening requires clinicians' strong professional knowledge, which greatly limits the early screening of cervical cancer in mass.

With the popularization of artificial intelligence, rapid discrimination by computer-aided diagnosis systems has become an effective means to solve the current dilemma of cervical cancer screening. The research on HPV site integration and the algorithm model corresponding to gene sequencing results and the classification diagnosis of cervical lesions are under continuous development. In addition, cytology and colposcopy visual examination, which focus on image processing, are well established in the application of deep learning, showing good performance on specific datasets [43, 44].

Due to the influence of various factors such as the dataset and the construction of classification standards, there is a certain one-sidedness in comparing the three types of research studies only from the accuracy. Some studies have carried out multimodal deep learning algorithm exploration on three types of data and finally found that the overall accuracy rate is better than that of the single-modal data. It can be seen that the three types of data play a certain value in the algorithm research for cervical lesion analysis. However, for early screening, blindly pursuing high accuracy and using multimodal examination will inevitably lead to a waste of resources. Therefore, it is the joint effort of researchers and clinicians to adopt appropriate computer-aided screening methods in specific environments.

This paper proposes a fusion method of Vision Transformer and DenseNet161 to classify cervical lesions in colposcopy images. In the experiment, acetic acid images, which are the most critical for clinical diagnosis, were used to train Vision Transformer and DenseNet161 by the fivefold cross-validation method, then, the fivefold prediction results corresponding to the two models were fused by weights, and finally, the fusion results are averaged to obtain the final lesion category. The results show that this fusion method improves the four-category classification accuracy of cervical lesions in colposcopy images to a certain extent.

In the experimental stage, we compared the model with several models that are currently widely used in the field of CV and found that the Vision Transformer alone is not ideal for classifying cervical lesions in colposcopy images. But when it is fused with DenseNet161 for fivefold cross-validation decision fusion, it achieves the best prediction accuracy. Even in the comparison of several other evaluation indicators, it is better than the fusion effect of DenseNet161 and EfficientNetV2.

This experimental finding revalidates our concern about model correlation in the process of fusion. We guess that although the ACC of EfficientNetV2 training alone is better, when it performs decision fusion with DenseNet161, which is also a CNN structure, the information obtained is more consistent because of their high similarity in feature learning, and the final classification is more like superposition effect. On the contrary, Vision Transformer, which is used to deal with the field of NLP, is no longer dominated by the same convolutional layer and has a quite different correlation with the DenseNet161 model. The features of cervical lesions in colposcopy images are studied from different levels, so more dimensional feature information is obtained, and finally, the four-category classification accuracy of cervical lesions is improved when the two models perform decision fusion.

At the same time, according to the comparison of the F1 score, we are pleased to find that the fusion of Vision Transformer and DenseNet161 is more suitable for the classification of cervical lesions in colposcopy images and is slightly less affected by the imbalance between cervical lesions. Moreover, the fusion method has a higher detection rate and a lower missed diagnosis rate of the lesion category, which is more conducive to the application of clinical complex environments, effectively helping physicians to improve diagnostic accuracy and ensure patients' life and health.

However, we also found that both Vision Transformer and DenseNet161 are heavyweight models, which take a long time in training and learning and occupy a large memory. Therefore, according to the findings of this paper, we will consider using the lightweight Vision Transformer for research on the basis of ensuring the predictive performance to explore a more practical and effective classification and diagnosis model of cervical lesions.

## 6. Conclusions

This paper proposes a fivefold cross-validation decision fusion method of Vision Transformer and DenseNet161 to perform a more refined four-category diagnosis on colposcopy images. This method combines the feature information of two models with correlation differences, which effectively improves the four-category classification accuracy of cervical lesion classification. The results show that the overall performance of the method in this paper is better than that of other models in the field of CV for the classification of cervical lesions in colposcopy images, and it is more suitable for the clinical environment. This can help physicians improve diagnosis efficiency and accuracy and reduce the risk of patients developing cervical cancer to ensure their life and health.

## Figures and Tables

**Figure 1:** Category samples of clinical colposcopy images.

**Figure 2:** The overall scheme of the method.

**Figure 3:** Data preprocessing.

**Figure 4:** Prediction process of cervical images by Vision Transformer model.

**Figure 5:** Prediction process of cervical images by DenseNet161 model.

**Figure 6:** Confusion matrices of DenseNet161 with EfficientNetV2 and Vision Transformer. (a) DenseNet161 + EfficientNetV2. (b) DenseNet161 + Vision Transformer.

**Table 1:** Data distribution.

Items	Negative		LSIL		HSIL		Cancer		Total	
	Cases	Images	Cases	Images	Cases	Images	Cases	Images	Cases	Image
Train	151	510	159	552	281	1180	41	170	632	2412
Test	24	24	23	23	43	43	10	10	100	100
Total	175	534	182	575	324	1223	51	180	732	2512

**Table 2:** Definitions of evaluation indicators.

Evaluation indicators	Definition
ACC	(TP + TN)/(TP + FN + FP + TN)
SEN	TP/(TP + FN)
SPEC	TN/(TN + FP)
PPV	TP/(TP + FP)
NPV	TN/(TN + FN)
F1 score	2 × PPV × SEN/(PPV + SEN)

**Table 3:** Comparison results between this fusion model and other models.

Model	Classes	ACC	F1	PPV	SEN	SPEC	NPV
Vision Transformer	Cancer	0.6000	0.8350	0.8136	0.8600	0.9780	0.9846
	HSIL		0.6184	0.5726	0.6744	0.6210	0.7190
	LSIL		0.4366	0.4984	0.3912	0.8778	0.8282
	Negative		0.6018	0.6556	0.5584	0.9080	0.8674

ShuffleNetV2	Cancer	0.6040	0.7722	0.7892	0.7600	0.9780	0.9738
	HSIL		0.6076	0.5744	0.6466	0.6384	0.7062
	LSIL		0.4628	0.5486	0.4086	0.8986	0.8364
	Negative		0.6386	0.6284	0.6498	0.8790	0.8884

MobileNetV3	Cancer	0.6260	0.7910	0.7490	0.8400	0.9692	0.9824
	HSIL		0.6402	0.5960	0.6930	0.6456	0.7372
	LSIL		0.4686	0.5376	0.4176	0.8934	0.8370
	Negative		**0.6564**	**0.7052**	0.6166	**0.9184**	0.8840

EfficientNetV2	Cancer	0.6360	0.8160	0.8406	0.8000	0.9824	0.9780
	HSIL		0.6346	0.6218	0.6512	0.6982	0.7268
	LSIL		0.5446	0.6158	0.4956	0.9064	0.8584
	Negative		0.6390	0.6096	**0.6750**	0.8632	**0.8944**

DenseNet161	Cancer	0.6560	0.8672	0.8500	**0.9000**	0.9802	**0.9890**
	HSIL		0.6514	**0.6684**	0.6420	**0.7544**	0.7388
	LSIL		0.5666	0.5798	**0.5654**	0.8778	0.8724
	Negative		0.6486	0.6370	0.6666	0.8790	0.8938

Ours	Cancer	**0.6800**	**0.9000**	**0.9000**	**0.9000**	**0.9890**	**0.9890**
	HSIL		**0.6890**	0.6600	**0.7210**	0.7190	**0.7740**
	LSIL		**0.6050**	**0.6500**	0.5650	**0.9090**	**0.8750**
	Negative		0.6380	0.6520	0.6250	0.8950	0.8830

**Table 4:** Comparison fusion results of different models.

Model	*ω*_1_	*ω*_2_	ACC
MobileNetV3 + ShuffleNetV2	0.65	0.35	0.61
Vision transformer + ShuffleNetV2	0.9	0.1	0.61
Vision transformer + MobileNetV3	0.3	0.7	0.61
ShuffleNetV2 + EfficientNetV2	0.1	0.9	0.65
MobileNetV3 + DenseNet161	0.3	0.7	0.66
Vision transformer + EfficientNetV2	0.05	0.95	0.66
MobileNetV3 + EfficientNetV2	0.35	0.65	0.67
ShuffleNetV2 + DenseNet161	0.1	0.9	0.67
EfficientNetV2 + DenseNet161	0.4	0.6	0.68
Vision Transformer + DenseNet161	0.05	0.95	0.68

**Table 5:** Comparison fusion results of DenseNet161 with EfficientNetV2 and Vision Transformer.

Model	Classes	F1	PPV	SEN	SPEC	NPV
DenseNet161 + EfficientNetV2	Cancer	0.900	0.900	0.900	0.989	0.989
	HSIL	0.682	**0.667**	0.698	**0.737**	0.764
	LSIL	**0.637**	**0.667**	**0.609**	0.909	**0.886**
	Negative	0.625	0.625	0.625	0.882	0.882

DenseNet161 + Vision Transformer	Cancer	0.900	0.900	0.900	0.989	0.989
	HSIL	**0.689**	0.660	**0.721**	0.719	**0.774**
	LSIL	0.605	0.650	0.565	0.909	0.875
	Negative	**0.638**	**0.652**	0.625	**0.895**	**0.883**

**Table 6:** Clinical comparison results of 100 test images.

Model	Classes	ACC	F1	PPV	SEN	SPEC	NPV
Colposcopists	Cancer	0.6200	0.6660	0.5710	0.8000	0.9330	0.9770
	HSIL		0.6850	**0.8330**	0.5810	**0.9120**	0.7430
	LSIL		0.5160	0.4100	**0.6960**	0.7010	**0.8850**
	Negative		0.6340	**0.7650**	0.5420	**0.9470**	0.8670

Ours	Cancer	0.6800	**0.9000**	**0.9000**	**0.9000**	**0.9890**	**0.9890**
	HSIL		**0.6890**	0.6600	**0.7210**	0.7190	**0.7740**
	LSIL		**0.6050**	**0.6500**	0.5650	**0.9090**	0.8750
	Negative		**0.6380**	0.6520	**0.6250**	0.8950	**0.8830**

## Data Availability

The processed data required to reproduce these findings cannot be shared at this time as the data also form part of an ongoing study.
